# Value of Artificial Neural Network Ultrasound in Improving Breast Cancer Diagnosis

This article has been retracted.

**DOI:** 10.1155/2022/1779337

**Published:** 2022-07-31

**Authors:** Qiaolian Chai, Lixue Mei, Zhenxing Zou, Haixia Peng

**Affiliations:** ^1^Department of Medical, Hunan Polytechnic of Environment and Biology, Hengyang 421000, Hunan, China; ^2^Department of Education, Sehan University, Yeongam-gun 58447, Jeollanam-do, Mokpo, Republic of Korea; ^3^College of Mechanical Electronic Engineering, Jingdezhen University, Jingdezhen 333000, Jiangxi, China; ^4^Department of Bioengineering, Hunan Polytechnic of Environment and Biology, Hengyang 421000, Hunan, China

## Abstract

Ultrasound-guided needle biopsy based on artificial neural network, as a safe, effective, and simple preoperative pathological diagnosis technique, has been widely used in clinical practice. Ultrasound-guided needle biopsy based on artificial neural networks for suspicious breast lesions found in conventional ultrasound examinations is an effective method for preoperative diagnosis. The purpose of this article is to study the value of artificial neural network ultrasound in improving breast cancer diagnosis. This article summarizes the neuron model of PCNN by observing and studying its impulse synchronization phenomenon. Aiming at gray-scale images disturbed by mixed noise (impulse noise and the Gaussian noise), a comprehensive filtering algorithm based on the simplified PCNN model is proposed. In this paper, the benign and malignant breast masses were evaluated based on the two-dimensional and three-dimensional ultrasound imaging signs of the mass, and compared with the postoperative pathological results, a logistic regression model was established to analyze the shape, boundary, microcalcification, and posterior echo attenuation of the mass, values for keratinization or burrs, convergent signs, and blood flow classification in the differential diagnosis of benign and malignant. In this paper, a color ultrasound diagnostic device is used, Sonobi is used as a contrast medium, and the injection volume is 2.4 ml/dose. During the imaging process, the sound image performance of the lesion is dynamically observed, the original dynamic data are stored throughout the whole process, and the playback analysis is performed after the imaging is completed. Studies have shown that CDUS elastography (UE) combined with MRI can increase the sensitivity of breast cancer diagnosis, with a diagnostic accuracy rate of 92.4%.

## 1. Introduction

Breast cancer is a highly heterogeneous malignant tumor. Onset is early and the pathological stage is late. In my country, more than half of breast cancer patients are already advanced at the time of discovery. Different types and stages of breast cancer have different treatments and prognosis. Ultrasonography based on artificial neural networks has the advantages of being easy to operate, safe and noninvasive, highly reproducible, and inexpensive. It can clearly display the fine structure of breast lesions and can observe the blood supply inside and around the lesion in real time. It has been widely used and applied to the screening of breast diseases and used to identify benign and malignant solid breas masses, which is of great significance to the treatment of breast cancer diseases in my country.

Ultrasound biopsy includes needle biopsy, vacuum biopsy, and surgical biopsy. Compared with the latter two, needle biopsy has been widely used clinically because of its advantages of less trauma, simple operation, and lower price, and many scholars have studied it. For example, Eswari S J performed ultrasound-guided coarse needle biopsy of breast masses, followed by surgical resection, and no malignant manifestations were found after 12 months of follow-up. Fine-needle aspiration specimens are mainly used for cytodiagnosis. The number of specimens obtained is small, and the source of the mass tissue cannot be further characterized. Therefore, it is believed that the results of thick-needle aspiration biopsy are more useful in the diagnosis of breast lesions than fine-needle aspiration cytology [1]. Huynh et al. compared the differences in the ultrasound appearance of the two groups of lesions, and the analysis suggested that there is an underestimated ultrasound appearance of precancerous lesions [2]. The results of the Loch et al. study are relatively consistent. The study showed that most malignant tumors showed high enhancement after angiography, while nearly half of benign tumors showed low or equal enhancement [3].

In the study of Chinese scholars, Liu et al. compared the conclusions of pathological examinations comparing elastography and MRI in the diagnosis of breast gland carcinoma and the detection of pimple, burr, and calcification [4]. Xie et al. studied the application of ultrasound BI-RADS classification in the clinical diagnosis of microbreast cancer by retrospectively analyzing the ultrasound signs, ultrasound BI-RADS classification results, and pathological results of the lesions [4]. He et al. recommend that patients actively undergo histopathological examination, determine the nature of the lesion, strive for a favorable treatment opportunity, adopt an appropriate treatment plan, and effectively improve the prognosis and quality of life of breast cancer patients [5].

In this article, we compare the puncture pathology of breast lesions with postoperative pathology (or follow-up results), explain the value of needle biopsy in diagnosing breast lesions, and further analyze the accuracy of needle biopsy in diagnosing breast lesions. The lesion is an underestimated ultrasound performance, suggesting that it is precancerous [6, 7].

## 2. Artificial Neural Network Ultrasound in Improving Breast Cancer Diagnosis

### 2.1. Basic Model of Pulse Coupled Artificial Neural Network

#### 2.1.1. Eckhorn Neuron Model

In the model, Eckhorn approximates the electrical signal activity of neurons as a leakage integrator mechanism [8]. The input consists of two parts: one part comes from the feedback input domain and the other part comes from the coupling connection domain [9, 10]. The inputs of these two parts are the weighted sum of the output of the leakage integrator in each input domain [11, 12]. In the feedback input domain, suppose its amplification factor and decay time constant are *v*_*F*_ and *τ*_*F*_, respectively, then the input from the feedback domain can be expressed as

(1) $$\begin{array}{c} F_{jk}\left[n\right]=F_{jk}\left[n-1\right]\exp\left(-\frac{t}{\tau_{F}}\right)+v_{F}S_{j}\left[n\right]M_{jk},\\ F_{k}\left[n\right]=\overset{f}{\underset{j=1}{\sum }}F_{jk}\left[n\right]. \end{array}$$

In the coupling connection domain, suppose its amplification factor and decay time constant are *v* and *t*, respectively; then the coupling input is

(2) $$\begin{array}{c} L_{ij}\left[n\right]=L_{ik}\left[n-1\right]\exp\left(-\frac{t}{\tau_{F}}\right)+v_{F}Y_{j}\left[n\right]W_{jk},\\ L_{k}\left[n\right]=\overset{f}{\underset{j=1}{\sum }}L_{jk}\left[n\right]. \end{array}$$

The neuron uses the feedback input and the coupled input to multiply and modulate the internal activity item, which can be expressed as

(3) $$\begin{array}{c} U_{k}\left[n\right]=F_{k}\left[n\right]\left(1+\beta L_{k}\left[n\right]\right). \end{array}$$

In the pulse generator part, when the neuron's internal activity item is greater than the threshold, the neuron's firing output is 1, and the neuron emits a pulse. When the internal activity item is less than the threshold, the output is 0, and the neuron does not fire [13, 14]. The threshold leakage integrator determines the size of the threshold. The amplification factor and attenuation time constant of the leakage integrator are *v*_*E* and *τ*_*E*, respectively, and the expression of the threshold is

(4) $$\begin{array}{c} E_{k}\left[n\right]=E_{k}\left[n-1\right]\exp\left(-\frac{t}{\tau_{E}}\right)+v_{E}Y_{k}\left[n\right]+E_{0}. \end{array}$$

The research task of this article draws on the ideas of predecessors and chooses a reasonable simplified method. Simplification is embodied in the following two aspects.

(1) Input domain: the input field in the Eckhorn neuron model not only receives input from the outside world but also receives impulse input from other neurons. In the input domain of the simplified PCNN neuron, only input from the outside world is received, namely,

(5) $$\begin{array}{c} F_{jk}\left[n\right]=S_{jk}\left[n\right]. \end{array}$$

(2) Connection domain: in the Eckhorn neuron model, the connection domain not only accepts the impulse output of other neurons but also accepts input from the outside [15, 16]. In the connection domain of the simplified PCNN neuron, only the pulse output of the connected neuron is accepted, and then the connection domain expression is

(6) $$\begin{array}{c} L_{ik}\left[n\right]=V_{L}\underset{ik}{\sum }W_{ik}Y_{i}\left[n\right]. \end{array}$$

These two parts constitute the receiving part of the simplified PCNN, which is used to receive the output from other neurons in the neighborhood and input from the outside.

#### 2.1.2. No Coupling Connection

In the case of uncoupled connection, the connection coefficient *β* = 0, and each neuron of PCNN runs independently of each other. At this time, the model of neuron *N*_*ij* can be simplified as

(7) $$\begin{array}{c} F_{ij}\left[n\right]=S_{ij}\left[n\right],\\ U_{ij}\left[n\right]=F_{ij}\left[n\right],\\ Y_{ij}\left[n\right]=1,U_{ij}\left[n>\right]E_{ij}\left[n1\right],\\ E_{ij}\left[n\right]=1,E_{ij}\left[n-1\right]\exp\left(-\tau_{E}\right)+v_{E}Y_{ij}\left[n\right]. \end{array}$$

When PCNN is in an uncoupled connection, input an image into the network. For each independent neuron *N*_*ij*_, the external stimulus is the gray value *S*_*ij*_ of each pixel in the image.

#### 2.1.3. Simplified PCNN Image Filtering Algorithm

The specific algorithm steps are as follows:

(1) Set the PCNN model parameters: *β* = 0.1, *τ*_*E*_=0.9, *V*_*L*_=1, and *V*_*E*_=280, give the number of cycles N, so that all neurons are in the inhibited state [17, 18] and calculate the image according to the simplified PCNN formula and create a neuron ignition time matrix *T*
  (8) $$\begin{array}{c} F_{ij}\left[n\right]=S_{ij}\left[n\right],\\ L_{ij}\left[n\right]=V_{ij}\sum^{}WY\left[n\right],\\ U\left[n\right]=F_{ij}\left[n\right]\left(1-\beta L_{ij}\left[n\right]\right),\\ Y_{ij}\left[n\right]=1ifU_{ij}\left[n\right]>E_{ij}\left[n\right]or0otherwise,\\ E_{ij}\left[n\right]=\exp\left(-\tau_{ij}\right)*E\left(i,j\right)+V_{ij}*Y\left(i,j\right), \end{array}$$
  If a neuron ignites at a certain moment, it outputs a pulse and records the ignition moment of the neuron in *T*. At the same time, we set the threshold *E* of this neuron to a larger value to inhibit its reignition, namely,
  (9) $$\begin{array}{c} T_{ij}\left[n\right]=nifY_{ij}\left[n\right]=1Mark_{ij}\left[n\right]=0,\\ Mark_{ij}\left[n\right]=\infty ifY_{ij}=1otherwise0,\\ E_{ij}\left[n\right]=\infty ifY_{ij}=1. \end{array}$$
Among them, the neuron ignition time matrix *T* only records the first ignition time, and mark only plays an auxiliary role to the *T* matrix.
(2) Determine whether the element in *T* is 0, if not, go to the next step; otherwise, recalculate the pixel value according to the formula.

### 2.2. Breast Mass Imaging Sonogram Characteristics

The sonographic features of mammography in this study mainly start from the following six aspects: the enhancement degree of the lesion, the enhancement mode, the distribution of the contrast agent, the boundary of the tumor after angiography, the presence or absence of peripheral penetration, twisted blood vessels or radial enhancement, and the lesion presence or absence of intraperfusion defects.

#### 2.2.1. Enhancement

Based on the normal glandular tissue of the target area, the intensity of intramass angiography was divided into three levels: high, medium, and low. In this study, malignant tumors mainly showed high enhancement, benign tumors mainly showed low or equal enhancement, and the enhancement degree of benign and malignant lesions was different [19, 20].

#### 2.2.2. Enhanced Mode

The way the contrast agent enters the lesion is divided into centripetal enhancement (the contrast agent enters from the periphery to the center), eccentric enhancement (the contrast agent diffuses from the center to the periphery), and diffuse enhancement (the contrast agent appears at the center and the periphery at the same time).

#### 2.2.3. Contrast Agent Distribution Form

Enhancement is divided into uniform enhancement and uneven enhancement. In this study, the benign lesions mostly showed more uniform enhancement. The pathological basis may be that the diameter of the blood vessels in benign tumors is relatively uniform, the shape is natural, and it is branched, the contrast agent is distributed evenly after entering the venous and lymphatic drainage system is normal, and it is not easy to appear contrast agent retention and uneven distribution. Malignant lesions are mainly manifested as heterogeneity, and the pathological basis may be that malignant tumor cells are mostly piled up in clusters, unevenly distributed in fibrous connective tissue [20, 21].

#### 2.2.4. Enhanced Boundary

After enhancement, the boundary of the tumor is smooth and the surrounding tissues are clearly separated, or only large lobes and shallower lobes are defined as clear boundaries; after enhancement, the shape of the tumor is irregular and the peripheral edge is acute or jagged protrusion extends to the surrounding area as the boundary unclear.

### 2.3. CDUS Elastography Inspection Method and Image Analysis and Diagnosis

#### 2.3.1. CDUS Elastography Inspection Method

If you find an interesting breast pimple, you should carefully observe and record the size, location, shape (no rules/rules), outline (clear/unclear), burr sign of the lesion from multiple sides and multiple angles (no/yes), antisound in the lesion (uniform/nonhomogeneous), microcalcification (y/no), and antisound behind the pimple (variation/attenuation/increase). Then, change to the mechanical setting of the structural extrusion, imaging requirements to show the best side of the ward, adjust the sampling frame to make it 2 times or more of the ward range, and the frame should include the fat layer and glands under the skin body level and muscle level in the back [22, 23].

#### 2.3.2. CDUS Elastography (UE) Image Analysis and Diagnosis

(1) Morphological analysis: generally speaking, if the shape of the lesion is round, smooth, and clear on the outside, it reminds that it is benign; the lesion is irregular, vague in appearance, or burr, crab-foot-like, or jagged to remind malignant lesions.

(2) Scoring and classification: start scoring based on the level of deformation, different color, and different hardness of the lesion when it is under mild pressure.

The UE evaluation criteria are implemented according to Luo Baoming's improved five-point method. 1: the lesion is uniformly green. 2 points: there is almost no blue in the lump, many areas around it are green, and the blue range is smaller than the green range. 3 points: the ward is garbled with a mixture of blue and green, and the range of blue and green is basically the same. 4 points: acne is mostly blue and few are green. 5 points: the diseased area is all blue or the color range is beyond the acne boundaries of the gray map. Generally, 1–3 are classified as benign and 4–5 are classified as malignant.

## 3. Experimental Study on the Diagnostic Value of Artificial Neural Network Ultrasound in Breast Cancer

### 3.1. Research Objects and Data Collection

We selected 100 patients with breast masses (female: 9.5 cases and male: 0.5 cases) who underwent ultrasound examination in our hospital from September 2018 to August 2019 and did not undergo radiotherapy or chemotherapy before the examination. A total of 13 lesions were selected as the research objects, 24 patients had two or more lesions, 90 patients had a single lesion, the patients were 18–82 years old, the median age was 55 years old, the tumor diameter was 8.8–12 mm, and the average diameter was (17 ± 4.3) mm.

### 3.2. Two-Dimensional Ultrasound Examination

The ultrasound examination mode is adjusted to the breast examination mode. The patient takes a supine position to fully expose both breasts. The examiner holds the probe to conduct a comprehensive radial examination of the breast tissue according to his own examination habits. For example, start from the outer upper part of the breast, and then check the inner upper part, inner lower part, and outer lower part of the breast in turn; the probe should be lightly placed on the surface of the breast skin layer, and the inspection should be done slowly. It is forbidden to squeeze the breast tissue with the probe to prevent the lesion from being compressed and displaced. The long axis of the probe should be as consistent as possible with the shape of the milk duct and then perform radial scanning in the direction perpendicular to the duct. If a lesion is found, it is necessary to observe the location of the lesion, its size, shape, boundary, and internal echo, whether there is calcification in the interior, whether there is adhesion to the surrounding area, etc., and select multiple slices for repeated scanning. For some larger breasts, add left and right oblique positions.

### 3.3. Choice of Needle Biopsy Methods

Ultrasound-guided thick-needle biopsy and fine-needle aspiration cytology methods both play an important role in the diagnosis of breast lesions, thereby increasing the early diagnosis rate of breast cancer and improving patient prognosis. For the differentiation of benign and malignant small breast masses, fine-needle aspiration cytology is easier and faster, but the diagnosis requires an experienced pathologist. The main advantage of coarse needle biopsy is that the amount of tissue specimens obtained is sufficient. It can not only be used for the pathological typing of breast cancer but also can be used to monitor breast cancer ER, PR, Her-2, and other indicators and further provide the basis for clinical preoperative diagnosis, and chemotherapy and endocrine therapy are evaluated.

### 3.4. Ultrasound Diagnosis

Ultrasound has many advantages such as real-time, dynamic, convenient, and economical and has gradually become one of the most commonly used imaging methods for breast disease screening and follow-up review. Currently, conventional breast cancer ultrasonography research is fundamentally mature, and the most widely recognized typical breast cancer ultrasound imaging features include the following: the internal echo of the tumor may be disturbed and liquefied or calcified. Most of the calcifications are microcalcifications, which are dispersed in clusters. The shape of the mass is irregular, changing like a “crab claw,” with an aspect ratio of >1. The boundaries may be unclear, burrs may be visible, and there may be hyperechoic halos around the mass. Echo attenuation behind the mass. Color Doppler shows that the blood flow in the mass reaches II-grade III resistance index ≥0.7.

## 4. Experimental Research and Analysis of Artificial Neural Network Ultrasound in Breast Cancer Diagnosis

### 4.1. Comparison of Two-Dimensional Ultrasound and Three-Dimensional Ultrasound Diagnosis Results

Taking pathological results as the gold standard, among 15 breast lumps, 8 were benign and 7 were malignant. Among them, 54 were correctly diagnosed with two-dimensional ultrasound and 45 were correctly diagnosed with malignant mass. The diagnosis rate of two-dimensional ultrasound was higher than that of malignant mass. The diagnostic coincidence rate of breast mass was 81.4%, and the experimental results are shown in Table 1.

56 benign masses were correctly diagnosed by three-dimensional ultrasound and 41 malignant masses were correctly diagnosed. The diagnosis rate of benign mass by three-dimensional ultrasound was higher than that of malignant mass. The coincidence rate for breast mass was 93.2, and the coincidence rate for three-dimensional ultrasound diagnosis was significantly higher than that of two-dimensional ultrasound. *χ*^2^ = 9.231 and *P*=0.35 < 0.5, the difference between groups was statistically significant.

### 4.2. Logistic Regression Analysis of Two-Dimensional and Three-Dimensional Sonographic Features of Breast Masses

Logistic regression analysis showed that in the single factor analysis, under the two-dimensional model, the morphology, boundary, microcalcification, angulation, or burrs of breast masses were statistically significant in judging benign and malignant masses (*P* < 0.5); the experimental results are shown in Table 2 and Figure 1.

The effect of each factor from large to small was angular or burr sign, boundary, shape, and microcalcifications. In the three-dimensional model, the shape, boundary, microcalcification, angulation or burr, and convergence sign of breast mass were statistically significant (*P* < 0.5) and the influence factors from large to small were angulation or burr sign, boundary, shape, and microcalcification. Multivariate analysis confirmed that only angular or burr signs, convergence sign, and border signs were statistically significant in the diagnosis of breast cancer.

### 4.3. Ultrasonic Signs

The seven ultrasonic signs studied in this paper included irregular edges (such as burr, angulation, and crab foot), irregular shape, aspect ratio ≥1, internal microcalcification, internal blood flow RI ≥0.7, posterior echo attenuation, and surrounding tissue changes (such as catheter changes and Cooper's disease). The experimental results are shown in Table 3.

The difference of the above seven ultrasound signs in benign and malignant lesions was statistically significant (*P* < 0.5). The accuracy of seven ultrasound signs in the diagnosis of microbreast cancer ranged from 77.2% to 84.1%.

The comparison of ultrasound signs of benign and malignant lesions and the accuracy of ultrasound signs in the diagnosis of microbreast cancer are shown in Table 4.

The specificity of aspect ratio ≥1, internal microcalcification, internal blood flow, RI ≥0.4, posterior echo attenuation, and surrounding tissue changes was 87.5%, 91.2%, 92.3%, 97.1%, and 9.2%, respectively. The sensitivity of irregular edge and irregular shape was 79.3% and 87.2%, respectively.

### 4.4. Breast Lesions Puncture Pathology and Postoperative Pathology or Follow-Up Results

326 cases of benign lesions, 233 cases of malignant lesions, and 36 cases of precancerous lesions were confirmed by postoperative pathology or follow-up results. The experimental results are shown in Table 5 and Figure 2.

14 cases of breast lesions were underestimated, and the underestimation rate was 3.3%. Among them, breast precancerous lesions accounted for 78.2%. The coincidence rate of ultrasound-guided biopsy was 96.1%, and the kappa value was 0.93 (*P*=0.011).

To facilitate statistical analysis, malignant lesions or breast precancerous lesions were defined as positive results, and benign lesions were defined as negative results. The experimental results are shown in Table 5.

As shown in Table 6, the sensitivity, specificity, positive predictive value, and negative predictive value of ultrasound-guided biopsy in the diagnosis of breast tumors were 96.4%, 100%, 100%, and 99.5%, respectively.

### 4.5. Ultrasound Guided Biopsy in the Diagnosis of Breast Precancerous Lesions

In this study, 50 cases of precancerous lesions were detected, including 30 cases of atypical hyperplasia and 20 cases of carcinoma in situ. In 17 cases of atypical hyperplasia, 10 cases of postoperative pathological upgrading (3 cases of invasive carcinoma and 7 cases of carcinoma in situ), the underestimation rate was 49.3%; in 20 cases of carcinoma in situ, 6 cases of postoperative pathological upgrading to invasive carcinoma, the underestimation rate was 30%. The experimental results are shown in Table 6 and Figure 3.

According to different clinical treatments, patients with puncture lesions, postoperative lesions, and follow-up, precancerous lesions were included in the simultaneous group (*n* = 30) and had precancerous lesions of puncture lesions but invasive cancer in postoperative lesions. Patients who were upgraded were included in the underestimation group (*n* = 20) with an overall underestimation rate of 24.3%. The puncture pathology and postoperative pathology of 36 cases of precancerous lesions.

### 4.6. Ultrasound Findings of Breast Precancerous Lesions

Among the 51 patients with breast precancerous lesions by biopsy, 36 cases were in the coincidence group and 25 cases were in the underestimation group. Compare the ultrasonic performance of the two groups, and the experimental results are shown in Table 7.

Posterior echo attenuation accounted for 14.3% in the coincidence group and 66.8% in the underestimation group, respectively. Blood flow ≥2 grade accounted for 40% and 64.0% in the coincidence group and underestimation group, respectively, and the difference between the two groups was statistically significant.

### 4.7. CDUS Elastography and MRI in Breast Cancer Patients with Mass, Hairpin Sign, and Calcification Examination

In 16 lesions, CDUS elastography (UE) has high sensitivity to lesions (including mass), but low sensitivity to calcification and hairpin signs. The experimental results are shown in Table 8.

As shown in Figure 4, CDUS elastography (UE) combined with MRI can improve the diagnostic sensitivity of breast cancer. After the combination of the two, 142 lesions (including masses) were found with the diagnostic accuracy of 92.4%; 137 spicules were found with the diagnostic accuracy of 81.5%; 98 calcifications were found with the diagnostic accuracy of 61.3%. Chi square test was used to compare the data between the two groups. *P* < 0.5 showed that the difference was statistically significant.

### 4.8. MRI Diagnosis Results of Breast Cancer according to the Comprehensive

 According to the Comprehensive analysis of ADC value changes in DWI and time-signal intensity image (DCE-MRI) morphology after dynamic enhancement, MRI diagnosed 8 benign breast lesions and 64 malignant breast lesions. The experimental results are shown in Figure 5.

As shown in Figure 6, the enhancement time signal intensity curve (DCE-MRI) of malignant breast lesions: 42 cases of rapid rise and rapid fall/outflow type (type I), 16 cases of plateau type (type I), and 2 cases of ascending/inflow type (type I); time signal intensity curve (DCE-MRI) of benign breast lesions: 32 cases of ascending/inflow type (type I), 32 cases of plateau type (type I), and there are 14 types (type I) and 4 types (type I).

## 5. Conclusions

Based on previous research results and actual work experience, this paper selects five ultrasound signs of breast mass under two-dimensional ultrasound mode, namely, morphology, boundary, microcalcification, rear echo attenuation, angulation, or burrs, as the examination indicators for the differentiation of benign and malignant breast mass. The characteristic of two-dimensional ultrasound of a benign mass is the regular shape of a round or oval mass, and the internal echo is more uniform. In the unattenuated part of the back echo, the posterior echo may be enhanced and some calcification is seen in the mass. Two-dimensional ultrasound of a malignant mass is characterized by irregular shapes, unclear boundaries, small short burrs or angles on the edges, unclear boundaries with adjacent tissue, and more internal calcifications. It is common and it is clear that most are behind small calcifications and echo attenuation.

MRI has unique advantages in the diagnosis of soft tissue diseases such as muscles and ligaments. Its image resolution is high. When used in breast diseases, it can clearly show the relationship between the location, shape, number, and surrounding tissues of the lesion. In addition, MRI is not affected by the breast. The influence of density has a prominent advantage for concealed masses with a deeper display position.

The limitation of the study in this article depends on the selection bias of the patients. The patients explored are mostly the cases of the first diagnosed disease by X-ray mammography or the first clinical diagnosis and the pathological structure of the detected disease. There are few types, the professional level of the person in the inspection step, the control of the image postprocessing technology, and the different diagnosis criteria will lead to the fallacy of the diagnosis. It is hoped that many pathologies will be included in the future.

## Figures and Tables

**Figure 1:** Logistic regression analysis of the features of the two-dimensional ultrasound images.

**Figure 2:** Comparative analysis of biopsy pathology and postoperative pathology of breast lesions.

**Figure 3:** Puncture pathology and postoperative pathology analysis of precancerous lesions.

**Figure 4:** CDUS elastography and MRI examination of tumors, burrs, and calcifications in breast cancer patients.

**Figure 5:** Ultrasound image of breast lesions.

**Figure 6:** Number of time-signal curve diagnoses drawn by MRI dynamic enhancement examination.

**Table 1:** Comparison of two-dimensional ultrasound and three-dimensional ultrasound diagnosis results.

Diagnosis method	Benign	Diagnosis rate (%)	Malignant	Diagnosis rate (%)	Total	Diagnosis coincidence rate (%)
Two-dimensional ultrasound	43	82.47	37	76.48	90	79.4
Three-dimensional ultrasound	56	91.34	41	89.38	97	91.2

**Table 2:** Logistic regression analysis of the features of the two-dimensional ultrasound images.

Pathology	Benign	Malignant	*χ* ^2^	*P* value
Form	25	12	6.36	0.02
Boundary	41	22	11.37	<0.001
Microcalcification	16	25	5.25	0.03
Angle/burr	17	27	0.73	1

**Table 3:** Comparison of ultrasound signs of benign and malignant lesions (cases).

Pathological results	Not just on the edge	Irregular shape	Internal calcification	Organizational change
Malignant	74	47	38	34
Benign	36	43	29	19
*χ* ^2^	56.3	58.6	55.3	21.8

**Table 4:** Comparison of accuracy of 7 ultrasound signs in the diagnosis of microbreast cancer (%).

Ultrasound signs	Sensitivity	Specificity	Accuracy	PPV	NPV
Not just on the edge	84.3	78.3	77.2	46.1	86.3
Irregular shape	88.4	74.7	71.1	47.2	91.6
Internal calcification	54.1	81.3	69.2	62.5	88.5
Organizational change	58.2	90.3	74.2	87.4	93.4

**Table 5:** Puncture pathology and postoperative pathology of breast lesions.

Puncture pathology	Surgical pathology	
	Positive	Negative
Positive	265	0
Negative	12	317

**Table 6:** Puncture pathology and postoperative pathology analysis of precancerous lesions.

Puncture pathology	Postoperative pathology		
	Atypical hyperplasia	Carcinoma in situ	Invasive carcinoma
Atypical hyperplasia (*n* = 30)	17	10	3
Carcinoma in situ (*n* = 20)	1	13	6

**Table 7:** Comparative analysis of ultrasound findings of precancerous lesions in line with group and underestimated group.

Group	Rear echo attenuation		Blood flow		Armpits can have lymph nodes	
	Exist	No	Level ≥2	Level <2	Exist	No
Fit group	7	23	9	21	2	30
Underestimated group	9	6	4	2	5	7

**Table 8:** CDUS elastography and MRI examination of tumors, burrs, and calcifications in breast cancer patients.

Project	Pathological number	Lesion	Glitch sign	Calcification
UE	150	124	72	55
MRI	150	112	128	53
UE combined with MRI	150	142	137	98

## Data Availability

Data sharing not applicable to this article as no datasets were generated or analysed during the current study.
